The article "Mutations of KRAS, NRAS, BRAF, EGFR, and PIK3CA genes in urachal carcinoma: Occurence and prognostic significance" was published in 2016. Journal: Oncotarget.

# Mutations of KRAS, NRAS, BRAF, EGFR, and PIK3CA genes in urachal carcinoma: Occurence and prognostic significance

**DOI:** 10.18632/oncotarget.9828

**Published:** 2016-06-05

**Authors:** Orsolya Módos, Henning Reis, Christian Niedworok, Herbert Rübben, Attila Szendröi, Szász Marcell A., József Tímár, Kornélia Baghy, Ilona Kovalszky, Tomasz Golabek, Piotr Chlosta, Krzysztof Okon, Benoit Peyronnet, Romain Mathieu, Shahrokh F. Shariat, Péter Hollósi, Péter Nyirády, Tibor Szarvas

**Affiliations:** ^1^ Department of Urology, Semmelweis University, Budapest, Hungary; ^2^ Institute of Pathology, University of Duisburg-Essen, Essen, Germany; ^3^ Department of Urology, University of Duisburg-Essen, Essen, Germany; ^4^ 2nd Department of Pathology, Semmelweis University, Budapest, Hungary; ^5^ 1st Department of Pathology and Experimental Cancer Research, Semmelweis University, Budapest, Hungary; ^6^ Department of Urology, Jagiellonian University, Krakow, Poland; ^7^ Department of Pathomorphology, Jagiellonian University, Krakow, Poland; ^8^ Department of Urology, Rennes University Hospital, Rennes, France; ^9^ Department of Urology, Medical University of Vienna, Vienna General Hospital, Vienna, Austria; ^10^ Tumor Progression Research Group, Hungarian Academy of Sciences, Budapest, Hungary

**Keywords:** urachal carcinoma, urachal cancer, urachus, mutation, EGFR, Pathology Section

## Abstract

**Purpose:**

Targeted therapy represents an attractive alternative for rare tumors such as urachal carcinoma (UrC). The aim of this study was to assess the mutations of the most commonly affected 5 genes in the targetable EGFR-pathway in UrC and comapre their frequencies to those of found in urothelial and colorectal cancer.

**Materials and Methods:**

Mutational hot-spots of selected genes were tested in 22 UrC samples by pyrosequencing. Mutational patterns were compared to those published for colorectal and urothelial cancers. Furthermore, we sought correlations between mutations and clinicopathological and follow-up data.

**Results:**

We found 11 mutations in 10 of 22 (45%) patients. The most frequently mutated gene was *KRAS* (27%) followed by *BRAF* (18%) and *NRAS* (5%), while no mutations were detected in the *EGFR* and *PIK3CA* genes. No correlation was found between the mutation status and clinicopathological parameters (Sheldon/Mayo stage, tumor grade, metastases). Furthermore, none of the mutations correlated with progression-free or overall survival.

**Conclusions:**

The mutation pattern of UrC is more similar to colorectal than to urothelial cancer. However, the mutation characteristics of UrC seems to be unique suggesting that clinical decision-making for UrC cannot be simply adopted from urothelial or colorectal carcinoma. The high occurence of EGFR-pathway mutations warrants the testing for *KRAS* and *BRAF* mutations when considering anti-EGFR therapy in UrC.

The article "Mutations of KRAS, NRAS, BRAF, EGFR, and PIK3CA genes in urachal carcinoma: Occurence and prognostic significance" was published in 2016. Journal: Oncotarget.

## INTRODUCTION

The urachus, or median umbilical ligament, is a midline tubular structure stretching between the bladder and the umbilicus. It is a remnant of embryonic development which gradually degenerates after the fourth month of embryonic life [1]. If the regression is incomplete, the urachus may persist and give rise to various abnormalities including malignances. Urachal cancer (UrC) is a rare, but highly malignant entity accounting for < 1% of all bladder cancers and mostly detected in conjunction with its invasion to the urinary bladder [2]. Because of its low incidence, our knowledge on the biology of UrC is limited. The recommended treatment for non-metastatic UrC is partial cystectomy with the complete removal of umbilicus and umbilical ligament [3]. Because of its hidden anatomical location at least 30% of UrCs are diagnosed at progressed stages, when a surgical treatment is not possible. In these cases, the most frequently used treatment is chemotherapy. As large scale, prospective clinical studies can hardly be performed for such a rare malignancy, clinical evidence and clear recommendations are not available for the systemic treatment of UrC. Therefore, the current chemotherapeutic treatment of UrC is rather based on individual decisions. The most frequently used chemotherapeutic agents are cisplatin and 5-fluorouracil [4–5]. The sparse data available on the efficacy of chemotherapeutic treatment in progressed UrC suggests 5-FU-based treatments to be superior to platinum-based therapies [4–5]. However, using any of these therapies the survival of UrC patients remains poor, warranting the need for more effective treatments. In the lack of evidence-based recommendations, targeted therapies tailored to the genetic features of each UrC case may provide an alternative approach in order to rationalize therapy decisions. To date there are only few, however promising data on the efficacy of targeted therapies in UrC. Testa *et al.* reported a necrotic involution of the tumor and a significant improvement of abdominal pain in a UrC patient who was treated with second-line multikinase inhibitor (Sunitinib) [6], while Goss *et al.* observed a size regression of a UrC as a response to EGFR-inhibitor therapy with gefitinib (Iressa) [7]. Finally, a recent study reported a patient with lung metastatic UrC who was effectively treated with a monoclonal EGFR-inhibitor (cetuximab) for eight months [8].

Both developing from the cloaca, urachal and colorectal adenocarcinomas (CRC) display several similarities regarding their histological, immunohistochemical and molecular features [9–10]. Mutated intracellular domain of EGFR is a therapeutic target in several malignancies including CRC as EGFR-inhibitors can silence mutation-activated EGFR signaling [11]. EGFR has three main downstream pathways: (1) RAS-RAF-MAPK, (2) PI3K-AKT and (3) JAK-STAT pathway, which stimulate mitosis leading to cell proliferation and inhibition of apoptosis [12]. A number of mutations of these downstream pathways are able to impair anti-EGFR treatment [11]. Therefore, mutation analyses of the EGFR-pathway are widely used for guiding treatment decisions [11, 13].

The article "Mutations of KRAS, NRAS, BRAF, EGFR, and PIK3CA genes in urachal carcinoma: Occurence and prognostic significance" was published in 2016. Journal: Oncotarget.

The prevalence and prognostic significance of the mutations in genes of the EGFR pathway in UrC remain poorly understood. Therefore, we screened the most commonly affected mutational hot spots of *KRAS, NRAS, BRAF, EGFR* and *PIK3CA* genes in the largest set of UrC samples evaluated to date and correlated them with patients' characteristics and survival.

## RESULTS

### Follow-up characteristics

Postoperative tumor recurrence was detected in two cases, metastatic tumor progression in two cases and local recurrence together with distant metastatic progression in five cases. The median time from surgery to first progression was 18 months. At the time of data evaluation 14 of 22 patients were alive with a median overall survival time of 35 months.

### Occurrence of mutations

We analyzed the mutations of the most frequently affected mutational hot-spots of *KRAS, NRAS, BRAF, EGFR* and *PIK3CA* genes in 22 UrC samples.

Overall, 11 mutations in 10 of 22 (45%) patients were found. *KRAS* was the most frequently affected gene with 6 mutations (6/22; 27%), followed by *BRAF* with 4 mutations (4/22; 18%) and *NRAS* with one case (1/22; 5%) (Tables 1, 2). In one case co-occurrence of an *NRAS* and a *BRAF* mutation was observed. No mutations in the EGFR and PIK3CA genes were detected.

**Table 1:** Mutations

Gene	Exon	Codon	Spot change	Amino change		Gene	Exon
KRAS	2	12	c.35G>A	p.G12D	GGT --> GAT	Gly --> Asp	1/22
	2	12	c.35G>T	p.G12V	GGT --> GTT	Gly --> Val	1/22
	2	13					0/22
	3	59					0/22
	3	61	c.182A>T	p.Q61L	CAA --> CTA	Gln --> Leu	1/22
	4	146	c.437C>T	p.A146V	GCA --> GTA	Ala --> Val	2/22
	4	146	c.436G>A	p.A146T	GCA --> ACA	Ala --> Thr	1/22
	∑						6/22
NRAS	2	12, 13					0/22
	3	59					0/22
	3	61	c.183A>T	p.Q61H	CAA --> CTA	Gln --> His	1/22
	4	146					0/22
	∑						1/22
BRAF	15	600	c.1799T>A	p.V600E	GTG --> GAG	Val --> Glu	4/22
EGFR	18	719					0/22
	19	744-750					0/22
	20	768, 790					0/22
	21	858-861					0/22
	∑						0/22
PIK3CA	9	542, 545					0/22
	20	1047					0/22
	∑						0/22

The article "Mutations of KRAS, NRAS, BRAF, EGFR, and PIK3CA genes in urachal carcinoma: Occurence and prognostic significance" was published in 2016. Journal: Oncotarget.

**Table 2:** Mutation frequency in different cancers

Mutations	Urachal cc		Bladder adenocc		Bladder TCC		Colorectal cc	
	*N*	%	*N*	%	*N*	%	*N*	%
KRAS	6/22 ^*^	27	2/21 ^18^	10	10/234 ^29^	4	3410/8350 ^25^	41
	3/7 ^33^	43			3/105 ^30^	3	613/1487 ^26^	41
	1/5 ^18^	20			4/218 ^31^	2	124/277 ^19^	45
	1/7 ^36^	14			4/98 ^32^	4	92/194 ^27^	47
	2/9 ^8^	22			0/128 ^17^	0	71/164 ^28^	43
							119/276 ^21^	43
**Σ**	**13/50**	**26**	**2/21**	**10**	**21/783**	**3**	**4429/10748**	**41**
NRAS	1/22 ^*^	5			2/105 ^30^	2	17/644 ^37^	3
	0/7 ^36^	0			0/218 ^31^	0	14/282 ^19^	5
	1/9 ^8^	11			4/98 ^32^	4	7/194 ^27^	4
					0/128 ^17^	0	25/276 ^21^	9
**Σ**	**2/38**	**5**	**-**	**-**	**6/549**	**1**	**63/1396**	**5**
BRAF	4/22 ^*^	18			0/145 ^31^	0	1288/11955 ^35^	11
	0/7 ^33^	0			0/128 ^17^	0	18/243 ^19^	7
	0/7 ^36^	0					10/194 ^27^	5
	0/9 ^8^	0					26/164 ^28^	16
							22/276 ^21^	8
**Σ**	**4/45**	**9**	**-**	**-**	**0/273**	**0**	**1342/12832**	**10**
EGFR	0/22 ^*^	0	0/28 ^18^	0	0/21 ^15^	0	17/236 ^20^	7
	0/7 ^36^	0			0/75 ^16^	0	3/280 ^19^	1
	0/9 ^8^	0			0/128 ^17^	0	11/276 ^21^	4
**Σ**	**0/38**	**0**	**0/28**	**0**	**0/224**	**0**	**31/792**	**4**
PIK3CA	0/22 ^*^	0			61/257 ^41^	24	108/743 ^37^	15
	0/7 ^36^	0			19/105 ^30^	18	24/255 ^19^	9
	1/9 ^8^	11			37/218 ^31^	17	32/194 ^27^	16
					26/128 ^17^	20	50/276 ^21^	18
**Σ**	**1/38**	**3**	**-**	**-**	**143/708**	**20**	**214/1468**	**15**

* results of this study

### Correlation of mutations with the clinical and follow-up data

We found no correlation between mutation status and clinicopathological parameters (signet ring cell differentiation, presence of calcification, Sheldon stage, Mayo stage, tumor grade and the presence of lymph node or distant metastases). However, all KRAS mutations were present in non-metastatic cases (6/18), this correlation missed the significance level (*p* = 0.176 − Chi-test). Furthermore, no association was detected between mutations and progression-free (*p* = 0.949) and overall survival (*p* = 0.942) (Figure 1).

**Figure 1:** Kaplan-Meier survival curves

## DISCUSSION

In the present study, we analyzed the mutation patterns of the most commonly affected genes of the EGFR-signaling pathway in UrC. The observed mutation frequencies were compared to those of CRC and urothelial carcinoma. Furthermore, we sought correlation between the detected genetic alterations and clinicopathological and follow-up data. Our results revealed a unique mutational profile for UrC which shows more similarities to CRC than to urothelial carcinoma.

The EGFR signaling pathway represents an important therapeutic target in various cancers e.g. in metastatic CRC [11]. Regarding efficacy of anti-EGFR therapy in UrC we found only one early two studies. An early phase I study assessed the effect of the EGFR-inhibitor gefitinib (Iressa) in various progressed solid tumors including lung, breast, colon, cervix and ovary cancers as well as one case of lymph node positive UrC [7]. From the 28, 22 included cases in this study, four showed clinical evidence of response and the one with UrC showed the highest decrease in tumor size of 55%, which was accompanied by a biological response as shown by the decrease of Ki67 proliferation index in the post treatment tumor biopsy [7]. In a recent publication Collazo-Lorduy et al. reported cetuximab treatment to be effective for eight months in a patient with metastatic UrC bearing *EGFR* amplification and wild-type KRAS [8]. These promising data suggest that anti-EGFR therapy might be effective also in UrC.

The article "Mutations of KRAS, NRAS, BRAF, EGFR, and PIK3CA genes in urachal carcinoma: Occurence and prognostic significance" was published in 2016. Journal: Oncotarget.

Primary resistance to EGFR inhibitors is mostly related to the presence of wild-type EGFR, as these tumors often harbor mutations in other genes downstream of EGFR such as *KRAS* and *BRAF* [14]. *EGFR* mutations were found to be absent in urothelial and primary bladder ADC and was reported to be also rare in CRC [12, 15–21]. Our present analysis provided similar results in UrC, revealing no mutations in the EGFR gene.

In the last years it became increasingly evident that activating structural mutations in one of the downstream pathway members can lead to resistance to anti-EGFR therapies (such as cetuximab). One of the most commonly affected downstream pathway is the RAS-RAF-MAPK signal way. KRAS is a G-protein encoding proto-oncogene and a member of the RAS protein family. In contrast to wild-type RAS proteins, which are deactivated after a short time, mutated RAS proteins cause continuous activation of RAS signaling pathways also without the upstream stimulation of EGFR or HER1 receptor [22, 23]. The oncogenic activation of RAS signaling pathways leads to abnormal cell growth, proliferation and differentiation. A somatic missense mutation in codon 12 of the *KRAS* gene, results in a single amino acid substitution (Gly12Val) representing the most frequently occurring mutation in CRC [22]. Further, less frequent KRAS mutations were found in KRAS codon 61 and 146 present in 1.5% and 3.2% of cases [24]. These *KRAS* mutant cases were unlikely to benefit from anti-EGFR therapy. Therefore, determination of its mutations has a crucial role in characterization and therapy of CRC [23]. In contrast to CRC [19, 21, 25–28], *KRAS* mutations are rare in urothelial carcinomas and primary bladder ADCs (~5% and ~10% respectively) [17–18, 29–32]. In UrC, Sirintrapun *et al.* observed 3 of 7 (43%) cases present with *KRAS* mutation, while Alexander *et al.* found mutation in 1 of 5 UrC patients (20%) [18, 33]. In accordance, we found similar occurrence (27%) for *KRAS* mutation in our 22 patients. Based on these, *KRAS* mutations - similar to CRC but in contrast to urothelial carcinomas - seems to be frequent in UrC. However, 3 of the 6 KRAS mutations we observed were located at codons 61 and 146 which are rarely (< 5%) affected in CRC.

The article "Mutations of KRAS, NRAS, BRAF, EGFR, and PIK3CA genes in urachal carcinoma: Occurence and prognostic significance" was published in 2016. Journal: Oncotarget.

About half of the CRC patients with wild-type KRAS do not respond to anti-EGFR therapy [34]. In these cases, mutated *BRAF* gene - which is present in ~10% of cases - can affect response to anti-EGFR treatment [35]. *BRAF* mutations were found to be absent in urothelial carcinoma, while, to best of our knowledge, there are no available data on the occurrence of its mutations in primary ADC of the bladder [17, 31]. In the present analysis, we found *BRAF* mutations in 4 of 22 (18%) UrC cases, which frequency seems to be similar to that of in CRC. In contrast, others found no *BRAF* mutations in UrC [8, 33, 36]. Low case number of that study together with the relative low abundance of *BRAF* mutation might be the reason for this discrepancy.

*NRAS* activating mutations were also found to be associated with failure of anti-EGFR therapy. Our analysis revealed one single UrC with *NRAS* mutation (1/22, 5%), suggesting, that these mutations are rare also in UrC similar to those of CRC [19, 21, 27, 31] and urothelial carcinoma [17, 30–32] (5% and 1% respectively).

The *PIK3CA* gene is involved in, the PI3K pathway affecting fundamental processes such as protein synthesis and cellular growth, mediated by mammalian target of rapamycin (mTOR) and S6 kinase. *PIK3CA* mutations in CRC are associated with clinical resistance to EGFR-targeted monoclonal antibodies [38]. Another therapeutically relevant correlation between the *PIK3CA* mutation and treatment response is related to aspirin. Experimental results demonstrated, that the inhibition of cyclooxygenase-2 (COX-2) by aspirin also down-regulates PI3K signaling activity [39]. In accordance, *PIK3CA* mutant CRCs were found to benefit from adjuvant aspirin therapy in contrast to patients with wild-type *PIK3CA* gene [40]. We found no *PIK3CA* mutations in any of the analyzed UrCs. In contrast, both urothelial [17, 30–31] and colorectal cancers [19, 21, 27, 31] were reported to bear *PIK3CA* mutations with a probability of 15-20% (Tables 2, 3).

We found no significant correlation between the mutation status and clinicopathological parameters of UrC (signet ring cell differentiation, presence of calcification, Sheldon stage, Mayo stage, tumor grade and the presence of lymph node or distant metastases). *KRAS* mutations were present only in non-metastatic cases (6/18), however, this correlation missed the significance level (*p* = 0.176 − Chi-test). Furthermore, none of the mutations correlated with progression-free or overall survival. In contrast, Sirantrapun *et al.* recently analyzed *KRAS* and *BRAF* mutations in 7 cases of UrC and found a better survival in patients with mutated *KRAS* gene [33]. This observation, however, is in contrast to those made in CRC and lung adenocarcinoma where *KRAS* mutations were associated with adverse prognosis. Therefore, the observed favorable prognostic effect of KRAS in UrC seems rather to be a consequence of low patient numbers than a real prognostic effect.

The article "Mutations of KRAS, NRAS, BRAF, EGFR, and PIK3CA genes in urachal carcinoma: Occurence and prognostic significance" was published in 2016. Journal: Oncotarget.

Recent publications provided whole exome sequencing data in samples UrC patients. Singh et al. identified recurrent mutations in *NF1, APC* and *RNF43* genes suggesting the involvement of MAPK and Wnt/β-catenin pathways in UrC formation [36]. In accordance, a further study found mutations in the MAPK pathway in four of nine cases [8].

Our study has some limitations regarding the low number of analyzed cases. Because of the extreme low incidence of UrC, only multi-institutional efforts can help to reach statistically relevant sample sizes. Being aware of this problem, we collected samples from multiple university centers. However, despite our study is one of the largest to date with molecular analysis on UrC, we have to acknowledge the sample size is still low, which does not allow a reliable statistical analysis. Therefore, further analyses with larger patient numbers are needed to confirm our findings.

## CONCLUSIONS

Our comparison between the mutation patterns of UrC and CRC as well as urothelial carcinoma revealed both similarities and differences. On the one hand, *KRAS* and *BRAF* mutations occurred in UrC with similar frequencies as in CRC, in contrast to urothelial carcinoma, where both of these mutations are infrequent. On the other hand, unlike in CRC, *PIK3CA* mutations seem to be absent. Finally, *EGFR* and *NRAS* mutations are rare in all these three tumor entities. These data suggest that the molecular features of UrC are rather similar to CRC than to urothelial carcinoma. However, the mutation characteristics of UrC seems to be unique, suggesting, that clinical decision making regarding UrC cannot simply adopted from evidence that is based on colorectal or urothelial carcinoma. Furthermore, our data suggest that patients with metastatic UrC, who are being considered for an anti-EGFR antibody therapy, should be tested for the presence of *KRAS* and *BRAF* mutations prior to therapy.

## MATERIALS AND METHODS

### Clinical samples

Twenty-two formalin-fixed, paraffin-embedded (FFPE) UrC samples were retrospectively collected from four academic centers. Inclusion criteria were histologically confirmed urachal adenocarcinoma localized to the urachus fistula and/or bladder dome. Cases with metastatic and/or local invasion to the bladder from other (e.g. gastrointestinal) cancers were excluded.

The article "Mutations of KRAS, NRAS, BRAF, EGFR, and PIK3CA genes in urachal carcinoma: Occurence and prognostic significance" was published in 2016. Journal: Oncotarget.

Clinical data including age, gender, tumor localization, Sheldon/Mayo-stage, grade, lymph node status and presence of distant metastasis, details on treatment, tumor recurrence, progression and survival were obtained from the medical records and relevant offices.

The median patient age was 52 years (range: 32-77 years). Sixteen of 22 patients were men (female-to-male ratio: 1:2.7). In three cases signet ring cell morphology and in another three cases calcification was observed. We used both the Sheldon [42] and Mayo systems [3] for stage classification. According to the Sheldon staging system [14], 10 patients were categorized into Sheldon stage IIIA, 7 into IIIB, 1 into IIIC, 2 into IVA and 1 into IVB, while the distribution regarding to the Mayo-system [3] was as follows: 4x stage I, 10x stage II, 5x stage III and 7x stage IV (staging data from one patient was not available). At the time of diagnosis, 4 patients (18%) had lymph node or distant metastasis. Initial surgical treatment was partial cystectomy in 15, radical cystectomy in 5 and transurethral resection (TURB) in 2 cases. In the two patients who underwent TURB, cystectomy was performed within a few weeks following transurethral resection. Eleven patients underwent umbilectomy and 13 patients had lymphadenectomy. Six patients received chemotherapy (Tables 3, 1). No chemotherapy or radiation was performed before surgery in any of the cases. The study was performed in accordance with the ethical standards of the Helsinki Declaration and was approved by the local ethical committee.

**Table 3:** Patients' characteristics and KRAS, NRAS and BRAF mutations

Variables		Patients		KRAS	NRAS	BRAF
		*n*	%	*n*	*n*	*n*
Age	≤ 55	14	64	4	1	3
	> 55	8	44	2	0	1
Gender	male	16	73	2	1	4
	female	6	27	4	0	0
Histology	ADC with SRC	3	14	0	0	1
	ADC without SRC	19	86	6	1	3
Calcification	present	3	14	1	0	0
	absent	19	86	5	1	4
Sheldon Stage	I-II	0	0	0	0	0
	IIIA	10	45	2	1	2
	IIIB	7	32	4	0	1
	IIIC	1	5	0	0	0
	IVA	2	9	0	0	0
	IVB	2	9	0	0	1
	IVC	0	0	0	0	0
Mayo stage	I	4	19	1	0	0
	II	10	48	3	1	3
	III	5	24	2	0	0
	IV	2	9	0	0	1
	missing	1				
LN or distant meta at diagn.	N0/M0	18	82	6	1	3
	N + / M+	4	18	0	0	1
Initial surgical treatment	partial CE	15	68	5	0	3
	radical CE	5	23	1	0	0
	TURB	2	9	0	1	1
Umbilectomy	yes	11	50	4	0	2
	no	11	50	2	1	2
LND	yes	13	59	3	0	2
	no	9	41	3	1	2
Chemotherapy	yes	6	27	1	1	2
	no	16	73	5	0	2
Progression	local recurrence	2	9	1	1	1
	distant met	2	9	1	0	0
	both	5	23	2	0	1
	no progression	13	59	3	0	2

Abbreviations:

ADC – adenocarcinoma

*SRC – signet ring cell differentiation*^+^

CE – cystectomy

LND – lymph node dissection

The article "Mutations of KRAS, NRAS, BRAF, EGFR, and PIK3CA genes in urachal carcinoma: Occurence and prognostic significance" was published in 2016. Journal: Oncotarget.

### DNA isolation and mutation analysis

Tumor containing areas were marked on hematoxylin and eosin (HE) stained sections by a pathologist and careful macrodissection has been performed in order to reduce contamination with non-malignant tissue. DNA was isolated from the dissected tissue sample using the High Pure PCR Template Preparation Kit (Roche, Mannheim, Germany) according to the manufacturer's recommendation. Extracted DNA concentrations were measured by a NanoDrop ND-1000 Spectrophotometer V3.3 (Thermo Fisher Scientific, Wilmington, DE, USA). Isolated DNA samples were amplified by polymerase chain reaction (PCR) for 13 exons of the 5 selected genes (*KRAS* exons 2, 3 and 4; *NRAS* exons 2, 3 and 4; *BRAF* exon 15; *EGFR* exons 18, 19, 20 and 21 and *PIK3CA* exons 9 and 20) on an Applied Biosystems Veriti^TM^ 96 well Thermal Cycler instrument (Applied Biosystems, Foster City, CA, USA). PCR conditions are shown in Suppl. table 1. PCR amplification products were analyzed on a PyroMark Q24 analyzer (Qiagen, Hilden, Germany) with PyroMark Q24 Software 2.0. All mutations were confirmed in a second analysis by repeating the PCR and pyrosequencing steps from the same DNA sample. Pyrosequencing primers were designed to test codons 12, 13, 59, 61 and 146 for *KRAS*, codons 12, 13, 59, 61, 117 and 146 for *NRAS*, codon 600 for *BRAF*, codons 719, 744-750, 768, 790 and 858-861 for *EGFR* and codons 542, 545 and 1047 for *PIK3CA*. Primer sequences are listed in Suppl. table 2.

### Statistical analysis

Results were correlated with clinicopathological and follow-up data. Chi-squared test was used to evaluate the association between mutation status and clinicopathological parameters. The Kaplan-Meier method with log-rank test was performed to estimate overall and progression-free survival. Statistical analyses were performed using the SPSS software version 20.0 (SPSS, Chicago, IL). The statistical significance was set at *p* < 0.05.

## SUPPLEMENTARY MATERIAL AND TABLES





## References

[1] Zhang J, Wu J (2013). Options for diagnosis and treatment of urachal carcinoma. Asia Pac J Clin Oncol.

[2] Bruins HM, Visser O, Ploeg M, Hulsbergen-van de Kaa CA, Kiemeney LA, Witjes JA (2012). The clinical epidemiology of urachal carcinoma: results of a large, population based study. J Urol.

[3] Ashley RA, Inman BA, Sebo TJ, Leibovich BC, Blute ML, Kwon ED, Zincke H (2006). Urachal carcinoma: clinicopathologic features and long-term outcomes of an aggressive malignancy. Cancer.

The article "Mutations of KRAS, NRAS, BRAF, EGFR, and PIK3CA genes in urachal carcinoma: Occurence and prognostic significance" was published in 2016. Journal: Oncotarget.

[4] Siefker-Radtke A (2012). Urachal adenocarcinoma: a clinician‘s guide for treatment. Semin Oncol.

[5] Szarvas T, Módos O, Niedworok C, Reis H, Szendröi A, Szász AM, Nyirády P (2016). Clinical, prognostic and therapeutic aspects of urachal carcinoma - a comprehensive review with meta-analysis of 1010 cases. Urol Oncol.

[6] Testa I, Verzoni E, Grassi P, Colecchia M, Panzone F, Procopio G (2014). Response to targeted therapy in urachal adenocarcinoma. Rare Tumors.

[7] Goss G, Hirte H, Miller WH, Lorimer IA, Stewart D, Batist G, Parolin DA, Hanna P, Stafford S, Friedmann J, Walsh W, Mathews S, Douglas L (2005). A phase I study of oral ZD 1839 given daily in patients with solid tumors: IND.122, a study of the Investigational New Drug Program of the National Cancer Institute of Canada Clinical Trials Group. Invest New Drugs.

[8] Collazo-Lorduy A, Castillo-Martin M, Wang L, Patel V, Iyer G, Jordan E, Al-Ahmadie H, Leonard I, Oh WK, Zhu J, McBride RB, Cordon-Cardo C, Solit DB, Sfakianos JP (2016). Urachal Carcinoma Shares Genomic Alterations with Colorectal Carcinoma and May Respond to Epidermal Growth Factor Inhibition. Eur Urol.

[9] Gopalan A, Sharp DS, Fine SW, Tickoo SK, Herr HW, Reuter VE, Olgac S (2009). Urachal carcinoma: a clinicopathologic analysis of 24 cases with outcome correlation. Am J Surg Pathol.

[10] Paner GP, McKenney JK, Barkan GA, Yao JL, Frankel WL, Sebo TJ, Shen SS, Jimenez RE (2011). Immunohistochemical analysis in a morphologic spectrum of urachal epithelial neoplasms: diagnostic implications and pitfalls. Am J Surg Pathol.

[11] Dietel M, Jöhrens K, Laffert MV, Hummel M, Bläker H, Pfitzner BM, Lehmann A, Denkert C, Darb-Esfahani S, Lenze D, Heppner FL, Koch A, Sers C (2015). A 2015 update on predictive molecular pathology and its role in targeted cancer therapy: a review focussing on clinical relevance. Cancer Gene Ther.

[12] Ciardiello F, Tortora G (2008). EGFR antagonists in cancer treatment. N Engl J Med.

[13] Wang HL, Lopategui J, Amin MB, Patterson SD (2010). KRAS mutation testing in human cancers: The pathologist‘s role in the era of personalized medicine. Adv Anat Pathol.

[14] Ellison G, Zhu G, Moulis A, Dearden S, Speake G, McCormack R (2013). EGFR mutation testing in lung cancer: a review of available methods and their use for analysis of tumour tissue and cytology samples. J Clin Pathol.

[15] Chaux A, Cohen JS, Schultz L, Albadine R, Jadallah S, Murphy KM, Sharma R, Schoenberg MP, Netto GJ (2012). High epidermal growth factor receptor immunohistochemical expression in urothelial carcinoma of the bladder is not associated with EGFR mutations in exons 19 and 21: a study using formalin-fixed, paraffin-embedded archival tissues. Hum Pathol.

The article "Mutations of KRAS, NRAS, BRAF, EGFR, and PIK3CA genes in urachal carcinoma: Occurence and prognostic significance" was published in 2016. Journal: Oncotarget.

[16] Blehm KN, Spiess PE, Bondaruk JE, Dujka ME, Villares GJ, Zhao YJ, Bogler O, Aldape KD, Grossman HB, Adam L, McConkey DJ, Czerniak BA, Dinney CP (2006). Mutations within the kinase domain and truncations of the epidermal growth factor receptor are rare events in bladder cancer: implications for therapy. Clin Cancer Res.

[17] Cancer Genome Atlas Research Network (2014). Comprehensive molecular characterization of urothelial bladder carcinoma. Nature.

[18] Alexander RE, Lopez-Beltran A, Montironi R, MacLennan GT, Post KM, Bilbo SA, Jones TD, Huang W, Rao Q, Sen JD, Meehan K, Cornwell A (2012). Miravalle L KRAS mutation is present in a small subset of primary urinary bladder adenocarcinomas. Histopathology.

[19] Peeters M, Oliner KS, Parker A, Siena S, Van Cutsem E, Huang J, Humblet Y, Van Laethem JL, André T, Wiezorek J, Reese D, Patterson SD (2013). Massively parallel tumor multigene sequencing to evaluate response to panitumumab in a randomized phase III study of metastatic colorectal cancer. Clin Cancer Res.

[20] Metzger B, Chambeau L, Begon DY, Faber C, Kayser J, Berchem G, Pauly M, Boniver J, Delvenne P, Dicato M, Wenner T (2011). The human epidermal growth factor receptor (EGFR) gene in European patients with advanced colorectal cancer harbors infrequent mutations in its tyrosine kinase domain. BMC Med Genet.

[21] Cancer Genome Atlas Research Network (2012). Comprehensive molecular characterization of human colon and rectal cancer. Nature.

[22] Chen J, Huang XF, Katsifis A (2010). Activation of signal pathways and the resistance to anti-EGFR treatment in colorectal cancer. J Cell Biochem.

[23] Jimeno A, Messersmith WA, Hirsch FR, Franklin WA, Eckhardt SG (2009). KRAS mutations and sensitivity to epidermal growth factor receptor inhibitors in colorectal cancer: practical application of patient selection. J Clin Oncol.

[24] Imamura Y, Lochhead P, Yamauchi M, Kuchiba A, Qian ZR, Liao X, Nishihara R, Jung S, Wu K, Nosho K, Wang YE, Peng S, Bass AJ (2014). Analyses of clinicopathological, molecular, and prognostic associations of KRAS codon 61 and codon 146 mutations in colorectal cancer: cohort study and literature review. Mol Cancer.

[25] Adelstein BA, Dobbins TA, Harris CA, Marschner IC, Ward RL (2011). A systematic review and meta-analysis of KRAS status as the determinant of response to anti-EGFR antibodies and the impact of partner chemotherapy in metastatic colorectal cancer. Eur J Cancer.

[26] Mao C, Huang YF, Yang ZY, Zheng DY, Chen JZ, Tang JL (2013). KRAS p. G13D mutation and codon 12 mutations are not created equal in predicting clinical outcomes of cetuximab in metastatic colorectal cancer: a systematic review and meta-analysis. Cancer.

The article "Mutations of KRAS, NRAS, BRAF, EGFR, and PIK3CA genes in urachal carcinoma: Occurence and prognostic significance" was published in 2016. Journal: Oncotarget.

[27] Foltran L, De Maglio G, Pella N, Ermacora P, Aprile G, Masiero E, Giovannoni M, Iaiza E, Cardellino GG, Lutrino SE, Mazzer M, Giangreco M, Pisa FE (2015). Prognostic role of KRAS, NRAS, BRAF and PIK3CA mutations in advanced colorectal cancer. Future Oncol.

[28] Ahn TS, Jeong D, Son MW, Jung H, Park S, Kim H, Bae SB, Kim HJ, Jeon YW, Lee MS, Baek MJ (2014). The BRAF mutation is associated with the prognosis in colorectal cancer. J Cancer Res Clin Oncol.

[29] Ouerhani S, Bougatef K, Soltani I, Elgaaied AB, Abbes S, Menif S (2013). The prevalence and prognostic significance of KRAS mutation in bladder cancer, chronic myeloid leukemia and colorectal cancer. Mol Biol Rep.

[30] Serizawa RR, Ralfkiaer U, Steven K, Lam GW, Schmiedel S, Schüz J, Hansen AB, Horn T, Guldberg P (2011). Integrated genetic and epigenetic analysis of bladder cancer reveals an additive diagnostic value of FGFR3 mutations and hypermethylation events. Int J Cancer.

[31] Sjödahl G, Lauss M, Gudjonsson S, Liedberg F, Halldén C, Chebil G, Månsson W, Höglund M, Lindgren D (2011). A systematic study of gene mutations in urothelial carcinoma; inactivating mutations in TSC2 and PIK3R1. PLoS One.

[32] Jebar AH, Hurst CD, Tomlinson DC, Johnston C, Taylor CF, Knowles MA (2005). FGFR3 and Ras gene mutations are mutually exclusive genetic events in urothelial cell carcinoma. Oncogene.

[33] Sirintrapun SJ, Ward M, Woo J, Cimic A (2014). High-stage urachal adenocarcinoma can be associated with microsatellite instability and KRAS mutations. Hum Pathol.

[34] Wilson PM, Labonte MJ, Lenz HJ (2010). Molecular markers in the treatment of metastatic colorectal cancer. Cancer J.

[35] Chen D, Huang JF, Liu K, Zhang LQ, Yang Z, Chuai ZR, Wang YX, Shi DC, Huang Q, Fu WL (2014). BRAFV600E mutation and its association with clinicopathological features of colorectal cancer: a systematic review and meta-analysis. PLoS One.

[36] Singh H, Liu Y, Xiao X, Lin L, Kim J, Van Hummelen P, Wu CL, Bass AJ, Saylor PJ (2016). Whole exome sequencing of urachal adenocarcinoma reveals recurrent NF1 mutations. Oncotarget.

[37] De Roock W, Claes B, Bernasconi D, De Schutter J, Biesmans B, Fountzilas G, Kalogeras KT, Kotoula V, Papamichael D, Laurent-Puig P, Penault-Llorca F, Rougier P, Vincenzi B (2010). Effects of KRAS, BRAF, NRAS, and PIK3CA mutations on the efficacy of cetuximab plus chemotherapy in chemotherapy-refractory metastatic colorectal cancer: a retrospective consortium analysis. Lancet Oncol.

[38] Ogino S, Lochhead P, Giovannucci E, Meyerhardt JA, Fuchs CS, Chan AT (2014). Discovery of colorectal cancer PIK3CA mutation as potential predictive biomarker: power and promise of molecular pathological epidemiology. Oncogene.

The article "Mutations of KRAS, NRAS, BRAF, EGFR, and PIK3CA genes in urachal carcinoma: Occurence and prognostic significance" was published in 2016. Journal: Oncotarget.

[39] Kaur J, Sanyal SN (2010). PI3-kinase/Wnt association mediates COX-2/PGE(2) pathway to inhibit apoptosis in early stages of colon carcinogenesis: chemoprevention by diclofenac. Tumour Biol.

[40] Li P, Wu H, Zhang H, Shi Y, Xu J, Ye Y, Xia D, Yang J, Cai J, Wu Y (2015). Aspirin use after diagnosis but not prediagnosis improves established colorectal cancer survival: a meta-analysis. Gut.

[41] Kompier LC, Lurkin I, van der Aa MN, van Rhijn BW, van der Kwast TH, Zwarthoff EC (2010). FGFR3, HRAS, KRAS, NRAS and PIK3CA mutations in bladder cancer and their potential as biomarkers for surveillance and therapy. PLoS One.

[42] Sheldon CA, Clayman RV, Gonzalez R, Williams RD, Fraley EE (1984). Malignant urachal lesions. J Urol.

